# MKA: A Scalable Medical Knowledge-Assisted Mechanism for Generative Models on Medical Conversation Tasks

This article has been retracted.

**DOI:** 10.1155/2021/5294627

**Published:** 2021-12-23

**Authors:** Ke Liang, Sifan Wu, Jiayi Gu

**Affiliations:** ^1^Pennsylvania State University, PA 16801, USA; ^2^National University of Defense Technology, 410073, China; ^3^Nvidia, Shanghai 201210, China; ^4^TMiRob, Shanghai 201203, China

## Abstract

Using natural language processing (NLP) technologies to develop medical chatbots makes the diagnosis of the patient more convenient and efficient, which is a typical application in healthcare AI. Because of its importance, lots of researches have come out. Recently, the neural generative models have shown their impressive ability as the core of chatbot, while it cannot scale well when directly applied to medical conversation due to the lack of medical-specific knowledge. To address the limitation, a scalable medical knowledge-assisted mechanism (*MKA*) is proposed in this paper. The mechanism is aimed at assisting general neural generative models to achieve better performance on the medical conversation task. The medical-specific knowledge graph is designed within the mechanism, which contains 6 types of medical-related information, including department, drug, check, symptom, disease, and food. Besides, the specific token concatenation policy is defined to effectively inject medical information into the input data. Evaluation of our method is carried out on two typical medical datasets, MedDG and MedDialog-CN. The evaluation results demonstrate that models combined with our mechanism outperform original methods in multiple automatic evaluation metrics. Besides, MKA-BERT-GPT achieves state-of-the-art performance.

## 1. Introduction

Difficulty in seeing a doctor, long queuing time, and inconvenience of making appointments have long been hurdles facing patients when they try to access primary care services. To solve these challenges, many advanced artificial intelligence (*AI*) technologies [1–3] have been combined with healthcare to boost the availability of medical resources, such as applying pattern recognition methods on medical images [4, 5] and leveraging natural language processing (*NLP)* technologies to design medical chatbots [6, 7]. The medical chatbot is mainly aimed to offer the medical assistants including disease identification, self-reports based medical suggestions for drugs, foods and checks, and medical front desk service guiding the patient to suitable healthcare service department, etc [8, 9]. It has a significant potential to simplify the diagnostic process and relieve the cost of collecting information from patients. Besides, the preliminary diagnosis results generated by the model may assist doctors to make a diagnosis more efficiently.

As the core of the medical chatbot, different methods have been investigated recently. In general, typical methods can be divided into two types [10], including information retrieval-based methods and neural generative methods. As for the first type, the methods usually match the response from the user-built question and answer (Q&A) pool based on the dialogue context, which means it can only provide the response that occurred in the existing pool. In another word, the poor-quality pool will influence a lot on the response. The second type of methods usually takes the dialogue context history as input and generates the suitable response word by word. Compared to retrieval-based methods, neural generative methods are more intelligent and flexible, which is what we focus on in this paper.

Currently, different neural generative models are applied to medical domain, including *LSTM-based* models, *Transformer*, *GPT*, and *BERT-GPT*. However, none of them performs well on the medical domain, which is reasonable. Here is the fact that the doctor makes diagnosis not only based on their experiences but also on the medical knowledge learned from professional books, especially when they meet rarely seen symptoms or diseases. The training procedure of the models only imitates the learning procedure of the experiences but leaves out the learning procedure from books. However, few works are about how to effectively integrate the medical knowledge with the neural generative models. Besides, patients are usually asked to fill in the patient self-report before the conversation starts with the doctor in real-world scenario. There are two common questions in the patient self-report, including “which department do you want to go?” and “what kind of the disease or symptom do you have?” Previous medical neural generative models will either leave out the information or roughly concatenate the original context in the patient self-report with the conversation history. It may cause either information loss or redundancy problem for the methods.

To address the limitations, the objective of the paper is to propose a medical knowledge-assisted mechanism (*MKA*) to assist common neural generative models to achieve better performance for the medical conversation task. *MKA* is an effective and lightweight method to integrate the medical knowledge with neural generative models. The mechanism first introduces a medical knowledge generation module to generate the related medical knowledge, which generates the medical knowledge subgraph (MKG_sub_) generated from the patients' self-report. The designed knowledge graphs contain related medical knowledge for each patient, including 6 types of entities (i.e., *ϵ*_department_, *ϵ*_disease_, *ϵ*_symptom_, *ϵ*_food_, *ϵ*_check_, and *ϵ*_drug_) and 6 types of relations (i.e., *γ*_has−disease_, *γ*_has−symptom_, *γ*_need−drug_, *γ*_need−check_, *γ*_need−food_, and *γ*_no−food_). Then, the medical knowledge information is fed into the token processor together with the dialogue contexts. Within the token processor, all the tokens will be reorganized based on the specific token concatenation policy. Finally, the processed data will be taken by selected generative models for training. In summary, we make the following contributions:

1. The paper proposes an effective and lightweight mechanism to integrate the medical knowledge into different neural generative models, *MKA*. Besides, the specific medical knowledge graph is designed to store the medical knowledge. To the best of our knowledge, *MKA* is the first scalable work that can integrate the medical knowledge into all kinds of neural generative models, especially for large-scale pretrained model, such as *BERT-GPT*
2. To verify our method, we implement two models based on our mechanism, *MKA-Transformer* and *MKA-BERT-GPT*. The evaluation is carried out on 2 typical medical conversation benchmarks: MedDialog [11] and MedDG [12]. Our experiments show that the model combined with our method outperforms previous methods in multiple automatic evaluation metrics. Besides, the *MKA-BERT-GPT* achieves the best performance on the task

The paper will be separated into 5 parts.  Section 2 will present the existing works related to medical dialogue generation tasks.  Section 3 will explain the details of the proposed mechanism.  Section 4 shows the experiment results and the analysis of the results.  Section 5 concludes the advantages and disadvantages of our work and its potential future works.

## 2. Related Works

Recent research on medical chatbots focuses on natural language understanding which leverages different advanced natural language processing (*NLP*) techniques. In general, the medical dialogue methods can be divided into information retrieval-based methods and neural generative methods according to the types of the applied *NLP* techniques. The retrieval-based methods can be further classified into different subtypes, such as the entity inference [12, 13], relation prediction [14, 15], symptom matching and extraction [16, 17], and slot filling [18–20]. However, the retrieval-based methods are not so intelligent and flexible that they required a well-defined user-built question and answer (Q&A) pool, which can offer different potential response to different kinds of answer. In another word, the retrieval-based methods only predict the link between question and answers in the pool, instead of learning how to respond to different questions like the doctors. Therefore, the neural generative methods have drawn more and more attention.

Nowadays, there is merely research on developing neural generative methods on medical domain. As an emerging research direction, most of the existing researches focus on testing different neural generative models on the benchmark domain-specific datasets. To figure out well the generative tasks in *NLP*, Hochreiter and Schmidhuber first proposed long short-term memory (*LSTM)* [21], which inspires multiple *LSTM-based* models [22–24]. Later, with the proposal of *Transformer* [25], researchers start to leverage *Transformer* units into novel dialogue generation models [26, 27]. Then, a more accurate and faster mechanism *GPT* is proposed [28]; different large-scale dialogue generative models are developed based on it [29, 30]. Meanwhile, some of the works also attempt to combine the different units to develop novel methods, where the state-of-the-art model is *BERT-GPT* model [31, 32]. However, the existing generative models for medical domain only learn the experience knowledge from the training procedure; few works effectively integrate the medical knowledge with the generative models.

## 3. Methodology

In this section, we discuss the methodology of *MKA*, which is a scalable, effective, and lightweight mechanism to integrate the medical knowledge into neural generative models, especially for large-scale pretrained model, such as *BERT-GPT*.

As shown in Figure 1, our *MKA* consists of 3 parts, including the medical knowledge generation module, token processor, and neural generative model. The medical knowledge generation module is constituted by medical knowledge subgraph generator, topic detector, and medical knowledge extractor. It is aimed at generating related medical knowledge information tuple. The token processor is proposed to concatenate the medical knowledge information tuple with the dialogue context for each conversation turn. Besides, the neural generative model is leveraged for training and prediction. The details of each module will be illustrated in Sections 3.1, 3.2, and 3.3.

### 3.1. Medical Knowledge Generation Module

The medical knowledge generation module is proposed to generate the related medical knowledge information when the doctor handles a case. Within the module, there exist three parts, including medical knowledge subgraph generator, topic detector, and medical knowledge extractor. The medical knowledge subgraph generator first takes the patient self-report which contains the department and disease/symptom information described in Section 1 as input and generates the medical knowledge subgraph (MKG_sub_) based on a global medical knowledge base (MKG_base_). MKG_base_ can be treated as a container which contains all the required medical professional books, while MKG_sub_ stores the potential useful medical knowledge related to the specific case. Different questions will be asked in different turns for the multiturn conversation task. To reduce the redundant information, the topic detector inputs the patient question at *i*^th^ turn and infers what question topic it related to. With the question topic and MKG_sub_, the medical knowledge extractor will extract the related medical knowledge information tuple. The details of each part will be shown as follows.

#### 3.1.1. Medical Knowledge Subgraph Generator

Within the medical knowledge subgraph generator, the medical knowledge subbase can be generated from the medical knowledge base based on the medical-related information extracted from patient self-report. In this paper, the knowledge base is represented the knowledge graph (KG), which is constituted by entities and relations. Besides, it is formally defined as below:

(1) $$\begin{array}{c} \text{KG}=\left(E,R,G=E\times R\times E\right), \end{array}$$

where *ℰ* represents the set of entities (e.g., persons), *ℛ* represents the considered types of relations between entities (e.g., friendship between persons), and *𝒢* is a set of 3-element fact tuples where each tuple represents a factual relation between two entities.

Therefore, two kinds of the medical knowledge graph (MKG) are proposed, including the medical knowledge base (MKG_base_) generated based on [33] by removing the redundant information and medical knowledge subgraph (MKG_sub_). Both MKG_base_ and MKG_sub_ contain 6 types of entities and 6 types of relations as shown in Tables 1 and 2. The entity and relation types are decided based on the working experiences of the author for the common medical conversation topics.

According to the definition of the entity and relation types, MKG_base_ contains 26910 entities (i.e., 54 *ϵ*_department_, 8807 *ϵ*_disease_, 5998 *ϵ*_symptom_, 4870 *ϵ*_food_, 3353 *ϵ*_check_, and 3828 *ϵ*_drug_) and 158216 fact tuples regarding the different relations (i.e., 8844 *γ*_has−disease_, 5998 *γ*_has−symptom_, 59467 *γ*_need−drug_, 39422 *γ*_need−check_, 22238 *γ*_need−food_, and 22247 *γ*_no−food_).

As for MKG_sub_, it is specific for each case, which is generated based on Algorithm 1. Within the algorithm, two subgraphs, *G*_1_ and *G*_2_, are extracted from MKG_base_ to constitute MKG_sub_. *G*_1_ is the graph with the *ϵ*_department_ type entity *ϵ*_1_^∗^ as the root. Besides, it only contains *γ*_has−disease_ and *γ*_has−symptom_ two types of relations. *G*_2_ is the graph with the *ϵ*_*disease*_/*ϵ*_*symptom*_ type entity *ϵ*_2_^∗^ as the root. Besides, it may contain all kinds of types of relations except *γ*_has−disease_. For more details, see Algorithm 1.

Meanwhile, it is worth noting that we propose a way to calculate the distance for entity matching as shown in

(2) $$\begin{array}{c} \text{dist}\left(u,v\right)=\left[\alpha \;\beta \right]\times \left[\begin{array}{c} {\text{dist}}_{\text{Levenshtein}}\left(u,v\right)\\ {\text{dist}}_{\text{Hamming}}\left(u,v\right) \end{array}\right], \end{array}$$

where *α* and *β* are two hyperparameters. The distance takes advantage of both the Hamming distance [34] and Levenshtein distance [35]. It can not only care about the meaning of the tokens like the Hamming distance but also the position of the tokens like Levenshtein distance.

#### 3.1.2. Topic Detector

The medical knowledge is related to what medical topic the patient asks. As a preparation for medical knowledge extractor, the question topic should be determined first. The content in the topic set matches with the relation set (i.e., disease, symptom, drug, check, positive food, and negative food). Besides, the six key phrase sets (KPS) are built corresponding to six topics based on the users' experiences. It consists of some specific phrases related to the question topic. Based on it, the question detector is proposed as shown in Algorithm 2.

#### 3.1.3. Medical Knowledge Extractor

The medical knowledge extractor is aimed at extracting the related medical knowledge information tuples based on question topic and medical knowledge subgraph from the previous two parts. It extracts all entities with the specific entity type and connected with specific relation type in the subgraph. Besides, *ϵ*_1_^∗^, *ϵ*_2_^∗^ extracted from patient self-report will be directly appended into the tuple, since they are also useful medical knowledge extracted from the source. The details are shown in Algorithm 3.

### 3.2. Token Processor

Compared to general neural generative models just taking dialogue contexts as inputs, our model generates the related medical knowledge information tuple which will be also fed into the models. To achieve this goal, a token processor is proposed to reorganize the tokens based on the policy shown in

(3) $$\begin{array}{c} X={\text{MKI}}_{i}⊕{\text{DR}}_{i-1}⊕{\text{PQ}}_{i}=\left[{\text{MKG}}_{\text{sub}}\text{ Unseen Features}\right]⊕\left[\text{PSR Seen Features}\right]⊕{\text{DR}}_{i-1}⊕{\text{PQ}}_{i}=\left[\text{All the elements in MK}{\text{I}}_{i}\text{ except }\varepsilon_{1}^{*}\text{ and }\varepsilon_{2}^{*}\right]⊕\left[\varepsilon_{1}^{*}⊕\varepsilon_{2}^{*}\right]⊕{\text{DR}}_{i-1}⊕{\text{PQ}}_{i}, \end{array}$$

where *X* represents the sequence for neural generative models and PSR represents patient self-report. MKI_*i*_, DR_*i*−1_, and PQ_*i*_ represent the medical knowledge information tuple in *i*^th^ conversation turn, the doctor response in *i* − 1^th^ conversation turn, and the patient question in *i*^th^ conversation turn separately. Besides, *ϵ*_1_^∗^ and *ϵ*_2_^∗^ are corresponding *ϵ*_department_ and *ϵ*_disease_/*ϵ*_symptom_ entities generated in Algorithm 1.

### 3.3. Neural Generative Model

In this paper, the neural generative model takes a source sequence *X* = (*x*_1_, *x*_2_, *x*_3_, ⋯, *x*_*T*_) consisting of *T* tokens generated from Section 3.2 and generates the response *Y* = (*y*_1_, *y*_2_, *y*_3_, ⋯, *y*_*T*′_) of length *T*′ tokens. In general, the model maximizes the generation probability of *Y* conditioned on *X* : *p*(*y*_1_, *y*_2_, *y*_3_, ⋯, *y*_*T*′_ | *x*_1_, *x*_2_, *x*_3_, ⋯, *x*_*T*_) [8], and the objective function of the sequence-to-sequence generative models is defined as below. Besides, as for the multiturn conversation tasks, the doctor response at *i*^th^ turn will be fed into the model as the existing dialogue context for next turn.

(4) $$\begin{array}{c} p\left(y_{1},\cdots ,y_{T\prime }\;|\;x_{1},\cdots ,x_{T}\right)=p\left(y_{1}\;|\;x_{1},\cdots ,x_{T}\right)\overset{T^{\prime }}{\underset{t=2}{\prod }}p\left(y_{t}\;|\;x_{1},\cdots ,x_{T},y_{1},\cdots ,y_{t-1}\right). \end{array}$$

## 4. Experiments

### 4.1. Experiment Settings

Our approach is implemented in Python 3.7 and PyTorch 1.4.0. We implement two MKA-Diagen models, including MKA-Transformer and MKA-BERT-GPT. The neural generative models within them are trained with the default parameters in [11, 25]. The hyperparameters *α* and *β* in Equation (2) are set as 0.1 and -1, and the hyperparameter *δ* is set as 0.7. We perform all the experiments on the Matpool server with 11 GB NVIDIA GeForce RTX 2080 Ti. Our experiments were performed on Chinese MedDialog dataset [11] and MedDG [12] with the ratio 0.8 : 0.1 : 0.1 of training set : validation set : test set.

The MKA-Transformer and MKA-BERT-GPT were compared with the baseline models (i.e., Transformer and BERT-GPT) and another typical nonsequence to sequence GPT-based model [11]. We followed the automatic evaluation metrics on the datasets to evaluate the performance of our method, including perplexity, NIST-2,4 [36], BLEU-2,4 [37], METEOR [38], Entropy-4 [39], and Dist-1,2 [40]. The perplexity shows the language quality of the generated responses. NIST-n, BLEU-n, and METEOR measure the similarity between the generated responses and ground truth and Entropy-n and Dist-n measure the lexical diversity of generated responses based on n-gram matching. The model with better performance will have the lower value of perplexity, the higher value of the other metrics.

### 4.2. Experiment Results and Analysis

In this part, the experiment results are shown together with the in-depth analysis of the results. Tables 3 and 4 show the performance on the MedDialog-CN test set and MedDG test set separately. From the tables, we make the following observations.

#### 4.2.1. Ablation Analysis

Focusing on the comparison between MKA-Transformer and Transformer and the performance comparison between MKA-BERT-GPT and BERT-GPT, it is easy to extract Table 5. It is easy to observe that our mechanism improves the performance from all aspects on both two datasets. It means that our method is effective and scalable to be applied to different neural generative models and different datasets.

#### 4.2.2. Performance Comparison Analysis

Compared to the current state-of-the-art models, our MKA-BERT-GPT outperforms all the other methods. It achieves the lowest perplexity. It is because its baseline generative model, BERT-GPT, is pretrained on a large collection of corpora before training on the medical specific datasets. The pertaining procedure helps it to better understand the linguistic structure among words; meanwhile, the medical knowledge-assisted mechanism enables the model more learnable for medical conversation task. Meanwhile, as for the machine translation metrics (i.e., NIST-4, BLEU-2, BLEU-4, and METEOR), the performance of the MKA-BERT-GPT also is the best. It even overturns the performance comparison between BERT-GPT and Transformer. It indicates that our method highly improves the overlap between the generated response and the ground truth. Besides, although the MKA-BERT-GPT improves the value on diversity metrics (i.e., Entropy and Dist), the improvement is still minor. It indicates that our model cannot make a big breakthrough on the capability in generating diverse responses.

#### 4.2.3. Case Study Analysis

Tables 6 and 7 represent the generated response of the models on two examples in the MedDialog-CN and MedDG test set. Since the dataset contains some Chinese medical dialogues, the translation is provided as well as the raw contents. The response generated by *MKA-BERT-GPT* is clinically informative and accurate. It prescribes “gastrointestinal functional problem.” Meanwhile, it can offer the detailed suggestions with rich medical knowledge information such as what kind of vegetables and fruits is recommended. Besides, the language quality of all the models is great, since all the responses are readable. Besides, there are still some spaces for the further improvement. For example, the responses generated from the models are not that overlap with the ground truth. It is because the ground truth is a Chinese medical response, which contains the concept of “qi,” which is not that easy for a general model to understand and provide the response. However, the responses of *MKA-BERT-GPT* are still relatively reasonable and also mention the conclusion of “the blood flow is not smooth.”

## 5. Conclusions

In this paper, we propose a scalable medical knowledge-assisted mechanism (*MKA*) to assist general neural generative models, especially the large-scale pretrained model, such as BERT-GPT, to achieve better performance on the medical conversation task. The mechanism introduces a medical specific knowledge graph, which contains 6 types of medical-related information, including department, drug, check, symptom, disease, and food. Besides, it also leverages the specific designed token concatenation policy and neural generative models. The promising experiment results have proven our mechanism is effective and scalable to different generative models on different medical conversation datasets. Besides, it also shows that *MKA-BERT-GPT* has achieved the state-of-the-art performance based on multiple automatic evaluation metrics compared to other existing models. In the future, we plan to apply the graph neural networks to extract and predict the related medical knowledge based on the medical knowledge base. Besides, it is also worthwhile to carry out the research on leveraging the advantages of both information retrieve methods and the neural generative methods to build a powerful dialogue generation system.

## Figures and Tables

**Figure 1:** Framework of our scalable medical knowledge-assisted generative model, *MKA*. In the figure, the ellipsoids represent the modules inside of our method. The orange ellipsoids show the automatic and scalable medical knowledge generation module. The figure legend inside of medical knowledge subgraph is corresponding to the entity types and relation types shown in Tables 1 and 2.

**Algorithm 1:** Pseudocode of the medical knowledge subgraph generator.

**Algorithm 2:** Pseudocode of the topic detector.

**Algorithm 3:** Pseudocode of the medical knowledge extractor.

**Table 1:** Definition of entity types in medical knowledge graphs.

Entity type	Description
*ϵ*_department_	Entities for the clinical departments
*ϵ*_disease_	Entities for the diseases
*ϵ*_symptom_	Entities for the symptoms
*ϵ*_food_	Entities for the food
*ϵ*_check_	Entities for the drugs
*ϵ*_drug_	Entities for the checks

**Table 2:** Definition of relation types in medical knowledge graphs.

Relation type	Description
*γ*_has−disease_	Relations between *ϵ*_department_ entity and *ϵ*_disease_ entity
*γ*_has−symptom_	Relations between *ϵ*_disease_ entity and *ϵ*_symptom_ entity
*γ*_need−drug_	Relations between *ϵ*_disease_/*ϵ*_symptom_ entity and *ϵ*_drug_ entity
*γ*_need−check_	Relations between *ϵ*_disease_/*ϵ*_symptom_ entity and *ϵ*_check_ entity
*γ*_need−food_	Relations between *ϵ*_disease_/*ϵ*_symptom_ entity and recommended *ϵ*_food_ entity
*γ*_no−food_	Relations between *ϵ*_disease_/*ϵ*_symptom_ entity and not recommended *ϵ*_food_ entity

**Table 3:** Comparison of the models on MedDialog-CN, where the best results are in bold.

Model	Dialog-GPT	Transformer	BERT-GPT	MKA-Transformer	MKA-BERT-GPT
Perplexity	9.71	9.52	8.23	8.81	**8.04**
BLEU-2	5.21%	4.92%	4.88%	5.02%	**5.71%**
BLEU-4	1.83%	0.90%	0.97%	0.99%	**1.35%**
NIST-2	0.36	0.42	0.40	0.43	**0.44**
NIST-4	0.32	0.40	0.39	0.40	**0.43**
METEOR	12.32%	13.11%	12.83%	13.4%	**13.94%**
Entropy-4	13.73	13.51	13.8	13.72	**14.1**
Dist-1	0.02%	0.03%	0.03%	0.03%	**0.04%**
Dist-2	2.01%	2.02%	2.14%	2.11%	**2.22%**

**Table 4:** Comparison of the models on MedDG, where the best results are in bold.

Model	Dialog-GPT	Transformer	BERT-GPT	MKA-Transformer	MKA-BERT-GPT
Perplexity	8.53	8.52	5.98	8.41	**5.95**
BLEU-2	6.41%	6.30%	7.62%	6.62%	**8.09%**
BLEU-4	2.12%	2.08%	2.57%	2.40%	**2.87%**
NIST-2	0.38	0.37	0.42	0.39	**0.43**
NIST-4	0.35	0.35	0.39	0.38	**0.41**
METEOR	13.78%	14.32%	16.25%	14.88%	**16.63%**
Entropy-4	10.56	10.17	**13.38**	10.28	13.37
Dist-1	0.01%	0.01%	**0.02%**	0.01%	**0.02%**
Dist-2	1.72%	1.67%	**2.00%**	1.69%	**2.00%**

**Table 5:** Improvements of the models with MKA compared to the baseline model on MedDialog-CN and MedDG test sets.

Dataset	Model	Perplexity	BLEU-2,4	NIST-2,4	METEOR	Entropy-4	Dist-1,2
MedDialog-CN	MKA-Transformer	-0.71	0.10%, 0.09%	0.01, 0	0.29%	0.21	0.00%, 0.09%
	MKA-BERT-GPT	-0.19	0.83%, 0.38%	0.04, 0.04	1.11%	0.3	0.01%, 0.08%

MedDG	MKA-Transformer	-0.11	0.32%, 0.32%	0.02, 0.03	0.56%	0.11	0.00%, 0.02%
	MKA-BERT-GPT	-0.03	0.47%, 0.30%	0.01, 0.02	0.38%	-0.01	0.00%, 0.00%

**Table 6:** An example of generated responses on the MedDialog-CN test set.

Patient self-report		科室 department: 男科 andrology 疾病/症状 disease/symptom: 静索静脉曲张 varicose veins
Patient question 1		我很怕是高位结扎手术引起的附睾炎, 希望大夫能给我说说是怎么回事, 该怎么处理? I am very afraid that it is the epididymitis associated with the high ligation operation. I hope the doctor can tell me how to deal with it quickly.

Doctor response 1	Ground truth	中医药调理。 You can recuperate yourself with Chinese medicine.
	Dialog-GPT	手术部位不会引发附睾炎。 The surgical part does not cause epididymitis.
	Transformer	可能是近期没有充分休息, 免疫力下降。建议早点休息。 It may be that you do not have enough rest and cause the decrease on the immunity. It is recommended to sleep early.
	BERT-GPT	不要趴着睡觉, 影响伤口恢复。建议多休息。 Do not sleep on your stomach, which will affect the recovery of the wound. It is recommended to rest more.
	MKA-Transformer	可以吃营养的健康食品, 比如西兰花, 鸡蛋等, 同时注重卫生清洁, 每晚可以热敷缓解疼痛。 You can eat nutritious and healthy foods, such as broccoli and eggs; meanwhile, pay attention to your hygiene and cleanliness. You can heat the area around your wound every night to relieve yourself.
	MKA-BERT-GPT	不可以吃冷饮, 少吃辛辣刺激的食物, 影响伤口恢复。建议多吃蔬果类, 比如苹果。不要久坐不动, 少穿紧身裤。 Do not drink cold drinks, and eat less spicy food, which will affect the recovery of the wound. It is recommended to eat more fruits and vegetables, such as apples. Do not sit for a long time and do not wear tight pants.

Patient question 2		请问我这是附睾炎吗?或是什么?恳请大夫您为我指点!感谢。 Is this epididymitis? Or what? I hope you, the doctor, to give me some advice! Thanks!

Doctor response 2	Ground truth	局部气血不畅。 The flow of the blood and qi in the local area is not that smooth.
	Dialog-GPT	放宽心, 只是心理作用。 Relax, it is just a psychological effect.
	Transformer	只是术后伤口疼痛。 It is just that the wound is painful after the operation.
	BERT-GPT	常见血流不通问题。 It is the common problem about the blood.
	MKA-Transformer	可能是运动过量导致提睾肌过度收缩, 导致疼痛。 Excessive exercise may cause excessive contraction of the cremaster muscle. It will make you feel painful.
	MKA-BERT-GPT	血流不通, 建议过几天复查伤口恢复情况, 减轻心理负担。 The blood flow is not smooth. It is recommended to review the situation of the recovery of the wound after a few days. Besides, you need to reduce the psychological burden.

**Table 7:** An example of generated responses on the MedDG test set.

Patient self-report		科室 department: 肛肠科 anorectal branch 疾病/症状 disease/symptom: 便秘,便血 constipation, blood in the stool
Patient question 1		医生你好, 最近我大便总是很干燥, 而且有好几次大便之后, 发现有血, 我这个是什么情况? Hello, doctor. Recently, I have found my stools were very dry. Besides, there is blood inside of them if I poop for several times. What is wrong with me?

Doctor response 1	Ground truth	你好, 可能存在痔疮出血!但还是建议您做个肠镜! Hello, there may be bleeding from hemorrhoids! But it is still recommended that you have a colonoscopy!
	Dialog-GPT	你好, 这种情况容易出现内痔 Hello, this situation is prone to internal hemorrhoids.
	Transformer	你好, 考虑是痔疮。 Hello, it is considered as hemorrhoids.
	BERT-GPT	你好, 可能存在痔疮, 大便干结多久了? Hello, there may be hemorrhoids, and how long have the stools been dry and clumpy?
	MKA-Transformer	你好, 可能是痔疮, 建议您做个肠镜。 Hello, it may be hemorrhoids. It is recommended that you have a colonoscopy.
	MKA-BERT-GPT	你好, 可能是痔疮出血。此外, 建议您做个肠镜。 Hello, it may be bleeding from hemorrhoids. In addition, it is recommended that you have a colonoscopy.

Patient question 2		为什么我的大便是一粒一粒的, 很干燥, 像羊屎那样的? Why do my stools come in pieces, very dry, like sheep feces?

Doctor response 2	Ground truth	大便干结是功能性问题, 建议您多吃水果蔬菜, 养成排便习惯! The dry stool is a functional problem. It is recommended that you eat more fruits and vegetables to develop a bowel habit!
	Dialog-GPT	你好, 可能存在痔疮。 Hello, there may be hemorrhoids.
	Transformer	注意饮食, 多吃蔬菜水果。 Pay attention to your diet and eat more fruits and vegetables.
	BERT-GPT	建议您多吃蔬菜水果。 It is recommended that you eat more fruits and vegetables.
	MKA-Transformer	考虑是肠胃功能性紊乱, 建议您多吃水果蔬菜。 It is considered as a gastrointestinal dysfunction. It is recommended that you eat more fruits and vegetables, like apples.
	MKA-BERT-GPT	考虑是肠胃功能问题, 建议您多吃水果蔬菜, 比如梨, 香蕉。若还是这样的话建议您做个肠镜。 It is considered as the gastrointestinal functional problem. It is recommended that you eat more fruits and vegetables, such as pears and bananas. If this is still the case, it is recommended that you have a colonoscopy.

## Data Availability

The data used to support the findings of this study are included in the article.
